# Research on Construction and Risk Management of Operating Room Based on IoTs and Digitization

This article has been retracted.

**DOI:** 10.1155/2022/3776017

**Published:** 2022-02-08

**Authors:** Chen Zhang, Fengqian Jia, Wei Wang, Tiantian Xu

**Affiliations:** ^1^Surgical Anesthesia Center, Taikang Tongji (Wuhan) Hospital, Wuhan 430050, China; ^2^Surgical Anesthesia Department, Xiangyang Central Hospital, Affiliated Hospital of Hubei University of Arts and Science, Xiangyang 441100, China

## Abstract

This paper introduces the background and experience of the development of a digital operating room and designs the main functions of the digital operating room based on the Internet of Things, the impact on medical data in hospitals, and how to build the digital operating room to cope with the huge amount of data in the “data era.” The infrastructure of the digital operating room is described, as well as how to collect and transmit medical data, how to store large amounts of medical data, and how to analyze medical data and explore its hidden data value are also described. One hundred and four surgical patients from June 2020 to June 2021 were randomly selected for the study, and they were randomly and equally divided into 52 cases each in the control group and the observation group, with the control group implementing the management of conventional care methods and the observation group implementing information technology for care management, comparing the management effects of patients in both groups. The satisfaction of patients in the observation group was significantly higher than that of the control group (*P* < 0.05). The use of information technology to ensure the quality of care in the operating room not only can help patients recover early but also can help patients relieve the psychological pressure after surgery, thus improving the doctor-patient relationship, and has a significant application effect.

## 1. Introduction

The digital development of the operating room first began in the 1990s, and the initial concept was the integrated integration of operating room equipment. Nowadays, the digital operating room emphasizes more on the transmission and common early information, based on the high integration of operating room system and medical equipment and monitoring equipment [1] and based on the transmission network so that the operating room can quickly obtain the information in HIS, PACS, US'EMR, and other systems and other information from the outside world; meanwhile, it realizes the collection, transmission, recording, and sharing of surgical information (including video and audio information, monitor data, medical equipment information, etc.).

The digital operating room allows the closed operating room and the outside world to establish an information channel so that the operating room is truly integrated into the overall information construction of the hospital, realizing the exchange and communication between the operating room and other departments of the hospital and also realizing the all-round recording and reproduction of surgical information [2]. The digital operating room supports the following major functions: rapid access to intraoperative information: medical and nursing staff can quickly obtain the required surgery-related information; observation and learning: live or recorded surgeries can be observed and learned in the demonstration room; remote guidance/consultation: the surgical process is presented to experts in an all-round manner, and help from experts in other locations is obtained; medical evidence/scientific research: the stored surgical information can be used for medical data recording; and storage: the data, mainly surgical information, can be stored and effectively combined with electronic data from other information systems so that the data can be better used for data analysis [3].

In 2008, the state issued the “Eleventh Five-Year Plan for the Development of IC Card Applications in Health Systems,” proposing to strengthen the association of the medical industry with banks and other related departments and industries, promote the application of “one card” products in the medical field, expand the scope of medical services with IC cards [4], establish a medical and health supervision and traceability system with radio frequency identification (RFID) technology, and promote the construction of medical information systems.

In the ideal digital operating room, we use RFID technology to automatically identify the target object by using RF signal. Because RFID tag has the advantages of large data storage capacity, fast reading and writing speed, high data security, good physical performance, and strong scalability, RFID bar code technology is considered to be more suitable for identification and positioning system at home and abroad [5]. In recent years, the medical industry at home and abroad tries to gradually introduce radio frequency identification technology into the operating room management for patient and staff identification, surgical information verification, real-time monitoring of the management and verification of the use of surgical instruments, medical equipment and consumables, surgical drugs, blood transfusion, pathological specimens, the traceability of the handling of medical waste, and so on, which is essential for improving surgical safety, staff efficiency, operating room utilization rate, the management level of the operating room, and so on [6].

In this paper, we have introduced the background and experience of an IoT-based development of the digital operating room, designs of the main functions of digital operating room, the impact on medical data in hospitals, and the ways to build a digital operating room to cope with the huge amount of data in the “data era.” The infrastructure of the digital operating room is described, as well as how to collect and transmit medical data, how to store large amounts of medical data, and how to analyze medical data and explore its hidden data value are also described.

The remaining paper is arranged as follows. In Section 2, a brief literature review is presented specifically those that are tightly coupled to the proposed methodology. In Section 3, IoT-based development of the digital operating room, designs of the main functions of the digital operating room, the impact on medical data in hospitals, and how to build the digital operating room to cope with the huge amount of data in the “data era” are discussed. Experimental results and observations, which are collected, were presented both in textual and graphical formats in Section 4. Finally, concluding remarks are given in Section 7.

## 2. Related Work

Since the concept of “Internet of things” was first proposed in China in 2009, domestic Internet of things technology has appeared in operating room management [7]. The research on the application of IoT technology in operating rooms began to appear and was widely carried out, and the research was mainly distributed in tertiary hospitals with high medical level and a high degree of medical informatization in various provinces and cities. Through data extraction and systematic analysis of the existing literature, the scope of application of IoT technology in the operating room is roughly divided into the management of people and things, and most of the existing studies are about the application of RFID and 2D barcode [8].

A study was conducted on the application of IoT technology in the management of personnel, equipment, and items in the operating room [9]. Observing indicators include patient satisfaction, medical and nursing satisfaction, work quality scores, surgical opening on-time rate, surgical safety verification implementation rate, operator arrival on-time rate, registration time in and out of the operating room, preoperative preparation time, postoperative infection, equipment utilization rate, equipment usage time statistics rate, and equipment integrity rate. The results of the study show that the application of IoT technology for the management of personnel, equipment, and items in the operating room has significantly improved the satisfaction of patients, work quality, and efficiency.

The application of IoT technology to surgical patient information management has been studied and observed indicators including the incidence of abnormal surgical transfer handover and the accuracy of time node records [10]. A study was conducted on the application of IoT technology to surgical instrument management [11]. Observed indexes included: instrument cleaning qualification rate, instrument traceability success rate, correct label writing rate, instrument package loss rate, packaging error rate, expiration date management effect, staff satisfaction, instrument package single operation time, and so on. The results of the study showed that using IoT technology for surgical instrument information collection and traceability management can avoid manual work. The results of the study show that the use of IoT technology for information collection and traceability management of surgical instruments can avoid errors generated by manual data collection and improve the quality and efficiency of work in the operating room.

A study was conducted on the application of IoT technology to the safe doorway management in the operating room, and the observed indicators included: completion of registration time, information error rate, dress code violation rate, correct recovery rate of hand-washing clothes and pants, and so on [12]. The results of the study showed that the use of an RFID technology-based door control management system eliminated the need for manual verification of information, issuance of keys, and searching for closets and shoe lockers, which shortened the registration time and effectively avoided information errors. At the same time, the dress code is standardized, and the loss of hand-washing clothes and pants is reduced.

At this stage, many countries are actively promoting the development of IoT technology as a means to enhance their competitiveness; for example, the EU is focusing on stimulating a privately led IoT ecosystem; private companies in the USA are vigorously pursuing IoT strategies; Japan is maximizing the application of IoT technology based on existing complete infrastructure; and India has recently proposed an IoT policy based on public-private partnerships to establish its own IoT industry in India [13]. A study of previous literature reveals that compared to the current status of application of IoT technology in domestic OR management, foreign countries have developed from the mere application of products with RFID tags to the application of the entire RFID system and are continuously expanding the application of this system [14].

Automatic acquisition of time points of surgical activities and automatic identification of the status of the operating room have been achieved by applying sensor networks and RFID systems in the operating room, circumventing possible errors in manual recording and, at the same time, improving the efficiency of operating room management [15]. The application of IoT technology is used in the study of [16] to establish an integrated operating room information system that comprehensive collects and visualizes medical information to provide surgeons with various types of information quickly, efficiently, and securely during surgery.

Some experts believe [7] that the application of IoT technology in the management of operating rooms in its medical institutions tends to be common based on the perfect infrastructure construction of the whole society in Japan, and how to anonymize data and protect patient privacy while applying IoT technology to automate information collection is the focus of current research.

It has been shown [17] that the application of IoT technology to the various time points of surgical activity, combined with DRG (diagnosis-related groups) to calculate their associated revenue, thus enabling cost-benefit analysis of the operating room; reference [19] showed that the application of IoT technology can achieve real-time data collection and integrated control, thus simplifying risk management in open integrated operating rooms.

Currently, a lot of man power and funds have been invested in the existing research and practice of medical logistics management in domestic and foreign medical institutions, but there are only a few mature products that can be practically applied to the management of the operating department of medical institutions (e.g., operating room personnel, items, etc.). This project aims to form a complete IoT system for the operating room based on the existing research on RFID applications in actual clinical work and to optimize and manage the core resources of the operating department of medical institutions so that the operating room can be connected with things and people and can improve efficiency while complementing the safety verification of surgery, which can reduce the chance of medical errors due to mismanagement. The economic and social benefits of medical institutions can be greatly improved if these mature products, which are the result of research projects, are widely implemented in clinical settings. At the practical level, it can provide an applicable and practical tool for the evaluation of information technology platforms in hospital operating rooms; at the theoretical level, it can serve as a methodological discussion and provide a reference for future research, especially the construction of evaluation index systems.

## 3. Overview of the Internet of Things

The Internet of Things (IoT), that is, the Internet connected to things, based on the development and application of the Internet, refers to the combination of various information sensing devices, such as radio frequency identification tags, global positioning systems, infrared sensors, laser scanners and other devices with the Internet of Things to form a huge network, so as to achieve automatic identification, positioning, tracking and monitoring of objects [1], which is built on the basis of the Internet and is also an important symbol of the information era. The architecture of IoT technology is mainly composed of four parts: sensing layer, network layer, application layer, and public technology [18], as shown in Figure 2.

### 3.1. Perception Layer

The sensing layer is mainly used to collect physical events and data occurring in the physical world, including various physical quantities, identity information, and location information. The perception layer integrates sensor technology, intelligent networking technology, distributed information processing technology, and other technologies to monitor, sense, and collect various environmental or monitoring object information in real time through the collaboration of various integrated microsensors. The sensing layer uses embedded systems to process the information and transmits the sensed information to the base station nodes and access gateways in the access layer through random self-organized wireless communication networks in a multihop relay mode and finally reaches the client [5].

### 3.2. Network Layer

The network layer is built on the basis of the Internet, mobile communication network, wireless sensor network, and so on. In order to realize the demand for connecting things, the IoT network layer will use IPv6, 2 G/3 G/4 G, Wi-Fi, and other communication technologies comprehensively to realize the combination of wired and wireless, broadband and narrowband, sensing, and communication networks. The information sensed by the perception layer will be transmitted everywhere quickly, safely, and reliably, enabling long-distance and wide-range communication of items. The network layer bears a larger amount of data and faces higher quality of service requirements than the existing network, and the existing network is not yet able to meet the IoT needs, and the IoT needs to converge and extend the existing network and use new technologies to achieve more extensive and efficient interconnection functions [6].

### 3.3. Application Layer

The application layer completes the final interaction between items and people. The network layer and the perception layer collect the information of items on a large scale, summarize and unify it in the application layer for analysis and decision-making, and use it to support the information collaboration, sharing, and interoperability across industries, applications, and systems and improve the comprehensive utilization of information to serve people to the greatest extent. A key problem to be solved by the application layer of IoT is how to efficiently process the massive data coming from the network layer and extract effective information from it. The application layer mainly includes key technologies such as M2M technology, cloud computing technology, artificial intelligence, data mining, and middleware [7].

### 3.4. Public Technology

Public technologies do not belong to a specific level of IoT technology but are related to all three layers of the IoT technology architecture, including identification and resolution, security technologies, network management, and QoS management [5].

### 3.5. Analysis of the Evaluation System of Operating Room Information Management Based on IoT Technology

Through a large amount of domestic and foreign literature research, the evaluation system of information management combined with the workflow of the operating room and finally formed an evaluation system with environment informatization, personnel informatization, and object informatization as the first-level indicators, which is consistent with the purpose of the Internet of Things to achieve “human-human, human-object, and object-object information interaction.” In the process of establishing the evaluation index system, a combination of Delphi expert consultation and hierarchical analysis was applied. On the one hand, the experts were selected in terms of their titles, professional fields, and years of experience, and the authority coefficient of the experts showed that the experts involved in the consultation were generally more authoritative, so the consultation results were credible.

## 4. IoT-Based Digital Operating Room

### 4.1. Digital Operating Room Infrastructure Program

As shown in Figure 3, the subsystems are related to the digital operating room (such as nursing station, anesthesia department, management side, remote side, etc.). In order to achieve data interoperability between the two systems, adapters or interfaces are needed to complete the conversion of heterogeneous data and to avoid the impact of heterogeneity.

Teleconsultation and remote guidance are part of the digital operating room system but need to use the external network to establish connections with off-site specialists, so configure a firewall to achieve restrictions on access to the external network and protect the hospital intranet. Others, such as nursing stations, conference rooms, operating rooms, and so on, are also part of the digital operating room and can be directly connected to the transmission network, or an adapter or interface can be added for data structure conversion.

Each subsystem has a clear division of labor and supports the functions of the digital operating room by collaborating with each other. The overall system has good scalability and flexibility so that adding or subtracting a subsystem or modifying the functionality of a subsystem will not have a significant impact on other parts and can adapt to future changes in the hospital's needs.

### 4.2. Massive Medical Data Processing Based on Digital Operating Room

On the basis of the above architecture, the digital operating room needs to achieve the acquisition, high-speed transmission, efficient storage, and effective use of a large amount of medical data.

#### 4.2.1. Access to Medical Data

The basic goal of the digital operating room is to transmit medical data, such as surgical information from the operating room to the outside world for activities such as demonstration and observation, and to transmit patient information and remote guidance information from the outside world to the operating room to assist in surgery. Therefore, the acquisition of medical data is the key first step. The surgical information to be acquired includes video images (panoramic images, operative field images, demonstration room images, and remote images), audio (operating room audio and outside audio), bedside monitor data, and high-end medical equipment data. High-quality video and audio are captured with equipment such as operating field cameras, panoramic cameras, and microphones, and medical data are collected from devices such as bedside monitors and medical devices with the help of conversion equipment and connected to integrated terminals for centralized processing. In addition, in order to better reproduce the scenes in the operating room, multiple types of video and audio as well as medical information can be collected and displayed in a synchronized manner so that the viewer can obtain a full range of data from the operating room at a certain point in time.

#### 4.2.2. Transmission of Medical Data

The digital operating room is based on the transmission network to achieve data transmission, can use the P network (the hospital already that has the P network can be used) or optical fiber for high-speed data transmission, in order to complete a large amount of data transmission tasks. The decoding and reading can be done at the receiving end. High-quality codec standards (e.g., H.264 and G.729) are used to achieve high compression ratios for high-speed transmission without affecting the quality of video, audio, and images.

Compared with the P-network transmission mode, the fiber optic mode has a faster speed, so it can be transmitted directly and quickly without compression, but it requires relaying fiber, which is costlier.

#### 4.2.3. Storage of Medical Data

With the development of digital operating rooms, the amount of data that needs to be stored such as surgical information is also increasing; the rapid growth of the medical data scale is inevitable; and the era of massive medical data is slowly coming. Therefore, a storage network consisting of multiple storage devices is needed to support the storage and reading of massive data while ensuring high scalability to cope with future changes. Considering the characteristics of the hospital, SAN or PSAN can be used to structure the storage network. PSAN, for example, is based on P network construction, which connects servers and one or more storage devices through a dedicated storage network to build a storage system and is a high-performance storage method. PSAN is based on iSCS technology; the SCS protocol is completely encapsulated in the P protocol to achieve efficient access to data. The overall access speed of PSAN depends on the network bandwidth, and it has a good transmission performance based on Gigabit Ethernet.

A simple PSAN storage network schematic is shown in Figure 4; each storage device can be used to store specific data; when the storage capacity is insufficient, simply add storage devices, without changing the storage structure. The server is used to implement specific storage and reading operations on the data. When the application side sends out data storage or reading operations, the server will operate accordingly, storing data in the storage device or reading the required data from the storage device. In addition, PSAN also supports data backup and remote disaster recovery to ensure the security of data.

#### 4.2.4. The Use and Value of Medical Data

The digital operating room system collects and stores medical data in the operating room, and the collected data can be used for various applications such as demonstration and learning, remote instruction, conference discussion, and medical evidence.

Compared with ordinary data analysis, the analysis of medical data has certain special features, including the diversity of medical data, such as text, images, audio, and video, and medical data often have a certain degree of time. Therefore, we can analyze the data with the help of a timeline, for example, linking the whole process of patients from consultation to hospitalization and surgery to discharge based on the timeline, sorting and aggregating patients with the same disease or surgery, and then analyzing and summarizing them. In addition, we can also choose to use data warehousing and data mining technology; first use ETL tools for data processing of data sources, combining data from different information sources, cleaning and filtering to ensure the quality of the data and finally storing in the data warehouse; and then use data mining tools for hidden value mining [5].

Data analysis of large amounts of medical data can help hospitals by providing information that is not intuitively available. For example, we can collect information on all procedures that take longer than expected or have abnormalities and identify the causes of the abnormalities that may cause the procedure to take longer than expected or cause abnormalities; we can categorize and analyze certain problems that are likely to occur during a certain type of procedure so that we can provide answers to specific questions during the demonstration; we can analyze the basic information about the patient and the difficulties during the procedure so that patients with a specific condition may suggest a difficult surgical point.

## 5. Information and Case Studies

### 5.1. Materials and Methods

One hundred and four surgical patients from June 2020 to June 2021 were randomly selected for the study: 45 patients for bone tissue surgery, 20 patients for reproductive system surgery, 15 patients for circulatory system surgery, and 24 patients for respiratory system surgery. They were randomly and equally divided into control group and observation group of 52 cases each: the average age of the control group was 35 years old; and the average age of the observation group was 34 years old. The difference between the general data of the two groups was not significant (*P* > 0.05), and the results were comparable [9].

The control group was managed in a conventional mode, following medical advice and using appropriate care measures for patients.

The observation group adopted a management model based on information technology.

1. Patients who need surgery are often worried that the surgery will be unexpected. Nursing staff need to explain to patients about surgery and self-care methods to relieve patients' fear and other negative emotions.
2. Check the patient's information in a timely manner and check whether there is any family history and so on.
3. Preoperative surgical planning and contingency planning should be done to ensure that surgical support is in place.
4. For intraoperative care, the nursing staff should be patient with patients who need to be accompanied to relieve their psychological pressure.
5. After surgery, dress the wound and change the medication in a timely manner, care for the patient, ask if there is discomfort, and inform postoperative precautions.
6. Make postoperative follow-up visits: 3–6 d after surgery, the patient's recovery situation was visited, and appropriate guidance was given.
7. Adopt information technology to guide patients' postoperative care behaviors, centralize patient management through the WeChat group, publish suggestions that can help patients' physical recovery in the WeChat group and so on, and supervise timely feedback from patients who have completed relevant care behaviors [3–4].

Patients in both groups were classified as very satisfied, satisfied, and unsatisfied, with 80–100 being very satisfied, 60–79 being satisfied, and <60 being unsatisfied.

SPSS 20.0 statistical software was selected for data processing, and *P* < 0.05 indicated that the differences were statistically significant.

### 5.2. Results

The results showed that the patients in the observation group were significantly more satisfied than the control group (*P* < 0.05; see Table 1).

### 5.3. Network Performance

The impact of the digital operating room on hospital medical data refers to medical and health-related data. Under the traditional model, these medical data are recorded and stored in different ways, including paper records, electronic records, and so on, and stored in different places, which cannot effectively process and use a large amount of data.

The information construction of the hospital stores most of the medical data in the form of electronic archives, which improves the management and use efficiency. As shown in Figure 5, the stability of Internet of Things operating room network communication and the development of digital operating rooms make the recording and use of hospital medical data go one step further. The digital operating room stores and records the operation information, operation process, and other medical data in the operating room in the form of electronic archives and image archives, solves the limitations of the traditional paper archives and electronic archives, develops from the static data of text and pictures to dynamic video and audio data, and organically combines with the basic information, case information, and examination information of patients. It realizes a comprehensive record of the process from patient diagnosis and treatment to admission and treatment to healthy discharge. The development of digital operating rooms helps hospitals record medical data more completely. At the same time, it also brings a large amount of medical data based on surgical information. These medical data may hide a large amount of information with important medical value.

As shown in Figure 6, the performance of different surgical tests is shown. The image streaming solution in this paper has image optimization technology to save transmission time and ensure image quality, so as to truly achieve real-time transmission of high-quality images. Develop telemedicine services and display images through high-definition screens. Doctors can timely judge the lesions in the images, then match the patients' oral symptoms to give medical treatment suggestions, and refer the patients to nearby and appropriate medical places, so as to save the suffering of patients in remote areas and make up for the dilemma of inadequate medical man power in rural areas. Telemedicine care technology can also be used to dynamically track patient data and give preventive care suggestions. With the aging of population structure, there is a large demand for medical services. At the same time, the treatment difficulty is increased due to the aging of patients. With the combination of smart technology and medical technology and the interconnection of medical equipment, the safety of surgical patients will be greatly improved, and a patient-centered operating room will be developed.

As shown in Figure 7, we investigated the satisfaction of five patients with the designed packing.

## 6. Discussion

The operating room is a special department of the hospital, and its management quality should be paid attention to. The implementation of information management not only can improve the management quality but also can improve the work efficiency of medical staff. Operating room information management includes the management of operating room rules and regulations, operation process, and medical staff work. The results show that the use of information technology can improve nursing satisfaction. The application of information technology has brought new changes to the management of the operating room. In short, the application of information technology can optimize the workflow of the operating room and improve the efficiency and standardization of the operation.

Under the automatic quality control system, the operation risk is effectively controlled; the support and guarantee are provided for the laboratory to arrange the operation and other normal operations; and the opening time of the operation is changed. At present, the operation arrangement only takes 1∼1.5 h, so the nursing supervisor has more time to pay attention to the safety of patients and the improvement of nursing quality [18]. It can be seen that information technology helps optimize the surgical process.

The operating area is a relatively clean area with high cleanliness requirements. It is necessary to record the relevant information of personnel entering and leaving the operating room. The use of information technology can effectively record the situation of personnel entering and leaving the operating room; monitor the cleanliness of clothing, badges, and surgical bags of operating personnel; realize the effective management of personnel inside and outside the operating area; realize the control, time, data, surgical information and other management of personnel entering and leaving the operating area; and realize the tracking management of relevant data paths. By effectively controlling the surgical dressing transferred from the clean area to the polluted area, the cleanliness of the surgical area is ensured [5]. On the other hand, the use of information technology effectively controls the time of personnel in the room. Medical services can directly contact relevant personnel through the remote query function, so as to improve the utilization of the operating room and provide more appropriate resources.

## 7. Conclusion and Future Work

With the continuous development of digital and information technology, the digital operating room will have more changes and greater significance. With the progress of science and technology, the digital operating room can realize higher quality data acquisition and processing and faster data transmission to deal with more and more surgical information and data. With the improvement of storage technology, the digital operating room can realize efficient access and management of massive medical data to support the application of different aspects of the hospital; At the same time, more and more powerful data analysis and data mining tools can also find more information that can help the hospital in a large amount of data and make the data create more value.

In addition, the future construction scope will also develop from the digital construction within a single hospital to the overall digital construction across regional hospitals. Many hospitals and medical institutions in the region will form a unified medical body, realize the assistance of large hospitals to small hospitals, share medical data such as operation information and patient information, and make digital construction play a greater value and role in medical undertakings on the basis of more and more comprehensive medical data.

## Figures and Tables

**Figure 1:** Digital operating room scene.

**Figure 2:** IoT technology architecture.

**Figure 3:** Digital operating room infrastructure construction plan.

**Figure 4:** Storage network diagram.

**Figure 5:** Stability of Internet of Things operating room network communication.

**Figure 6:** Performance of different surgical tests.

**Figure 7:** Surgical satisfaction of different patients.

**Table 1:** Comparison of patient satisfaction between the two groups (cases).

Group	Very satisfied	Satisfied	Dissatisfied	Total satisfaction (%)
Control group	22	15	15	71.15
Observation group	27	18	7	86.54
*P*				<0.05

## Data Availability

The data sets used and analyzed during the current study are available from the corresponding author upon reasonable request.
